# Predicting Osteopathic Medical Student Performance on the United States Medical Licensing Examination Step 2 Clinical Knowledge From Results of the Comprehensive Osteopathic Medical Licensing Examination Level 2-Cognitive Evaluation

**DOI:** 10.7759/cureus.19625

**Published:** 2021-11-16

**Authors:** Travis Smith, J. Bryan Carmody, Mark Kauffman, James Gnarra

**Affiliations:** 1 Emergency Medicine, Lake Erie College of Osteopathic Medicine, Bradenton, USA; 2 Pediatric Nephrology, Eastern Virginia Medical School, Norfolk, USA; 3 Pediatric Nephrology, Children’s Hospital of The King’s Daughters, Norfolk, USA; 4 Family Medicine, Lake Erie College of Osteopathic Medicine, Bradenton, USA; 5 Microbiology and Immunology, Lake Erie College of Osteopathic Medicine, Bradenton, USA

**Keywords:** undergraduate and graduate medical education, graduate medical education (gme), usmle step 2, comlex level 2, match, residency selection, comlex-usa, usmle

## Abstract

Background

To improve their standing in residency selection, many osteopathic medical students choose to take the United States Medical Licensing Examination (USMLE). Although scores on USMLE Step 1 and Level 1 of the Comprehensive Osteopathic Medical Licensing Examination (COMLEX-USA) are known to be highly correlated, scarce data exist on the association between COMLEX-USA Level 2-Cognitive Evaluation (CE) and USMLE Step 2 Clinical Knowledge (CK) scores. In this study, we aimed to determine the association between COMLEX-USA Level 2-CE and USMLE Step 2 CK scores and derive an equation to predict performance on USMLE Step 2 CK for applicants who have only taken COMLEX-USA.

Methodology

We reviewed COMLEX-USA Level 2-CE and USMLE Step 2 CK scores for all students at the Lake Erie College of Osteopathic Medicine from May 2020 to April 2021. Linear regression was used to evaluate the relationship between COMLEX-USA Level 2-CE and USMLE Step 2 CK scores.

Results

A total of 340 students took both COMLEX-USA Level 2-CE and USMLE Step 2 CK. There was a linear association between COMLEX-USA Level 2-CE and USMLE Step 2 CK scores such that every one-point increase in COMLEX-USA was associated with a 0.13-point increase in USMLE Step 2 CK score (standard error = 9.1; model R^2^ = 0.64).

Conclusions

Students or programs interested in predicting performance on USMLE Step 2 CK from performance on COMLEX-USA Level 2-CE can do so using the following equation: USMLE Step 2 CK = 0.13(COMLEX-USA Level 2-CE) + 163.5.

## Introduction

To graduate from an osteopathic medical school, the Commission on Osteopathic College Accreditation requires that students pass both the Level 1 and Level 2 Cognitive Examination (CE) of the Comprehensive Osteopathic Medical Examination (COMLEX-USA) [1]. The COMLEX-USA is the only examination accepted for the initial licensure of osteopathic physicians in all jurisdictions in the United States [2]. However, >60% of osteopathic medical students also choose to take at least some portion of the United States Medical Licensing Examination (USMLE) [3]. This is not done for graduation or licensure requirements but to enhance residency applications. USMLE scores are the most frequently cited factor among residency program directors in identifying applicants to interview [4]. This generates substantial pressure for osteopathic medical students to take the USMLE to increase their chances of matching in a competitive program or discipline [5,6]. This comes at a high cost to the student and hundreds of added hours studying for two different examinations.

Numerous studies have demonstrated a linear association between osteopathic medical student performance on the COMLEX-USA Level 1 and the USMLE Step 1 examinations [7-13]. However, both of these examinations will soon transition to pass/fail score reporting. Surveys of residency program directors in multiple specialties suggest that USMLE Step 2 Clinical Knowledge (CK) performance will assume a more significant role in residency selection [14-21]. Unfortunately for students and their advisors, data on the association between COMLEX-USA Level 2-CE and USMLE Step 2 CK performance are sparse: the few studies that have examined this topic use data that are around 10-15 years old [7] or have included only data from a single residency program [8,10]. Therefore, we sought to reevaluate and update the relationship between scores on the COMLEX-USA Level 2-CE and USMLE Step 2 CK examinations in a large sample of contemporary osteopathic medical students who are applying to multiple residency programs in various specialties.

## Materials and methods

Setting and participants

We reviewed the COMLEX-USA Level 2-CE and USMLE Step 2 CK scores for all students at the Lake Erie College of Osteopathic Medicine (LECOM) who took both exams during the testing cycle between May 1, 2020, and April 30, 2021. COMLEX-USA and USMLE scores were obtained from school records. This data included those who took both examinations as well as those who only took COMLEX-USA Level 2-CE. For students who took either exam more than once, performance on the first exam attempt was analyzed.

Statistical analysis

We calculated descriptive statistics (including median and interquartile ranges [IQRs] for performance on each test) for the study population. To evaluate the association between COMLEX-USA and USMLE scores, we performed simple linear regression. A two-sided significance level of 0.05 was set for all tests. All statistical analyses were performed using SPSS version 27 (IBM Corp, Armonk, NY, USA).

Ethical approval

Because the investigators received only deidentified paired score data from the campus registrar, the LECOM Institutional Review Board (IRB) determined this research to be IRB-exempt and waived the need for consent.

## Results

From May 2020 to April 2021, there were 552 LECOM students who took the COMLEX-USA Level 2-CE examination. Of these, 340 (61.6%) also took the USMLE Step 2 CK examination. Among all test-takers, the median COMLEX-USA Level 2-CE score was 578 (IQR = 510-640.5; range = 283-896). The median USMLE Step 2 CK score was 240 (IQR = 231.25-250; range = 194-281).

Students who took both the COMLEX Level 2-CE and the USMLE Step 2 CK exams scored higher on COMLEX-USA Level 2-CE than those who did not take both exams [median 604 (IQR = 538.5-665) vs. median 531 (IQR = 469.25-592); p < 0.001, Mann-Whitney U test]. Overall, 23/552 (4.2%) of students failed COMLEX-USA Level 2-CE, while 10/340 (2.9%) failed USMLE Step 2 CK. Two examinees failed both tests. Students who did not take USMLE Step 2 CK were more likely to have failed COMLEX-USA Level 2-CE than those who took both exams (20/212 = 9.4% vs. 3/340 = 0.9%; p < 0.001, chi-square test).

Pairs of COMLEX-USA Level 2-CE and USMLE Step 2 CK scores are shown in the scatterplot in Figure 1. There was a linear association between performance on COMLEX-USA Level 2-CE and USMLE Step 2 CK scores, with every one-point increase in COMLEX-USA Level 2-CE associated with a 0.126-point increase in USMLE Step 2 CK score (95% confidence interval (CI) = 0.116-0.137; p < 0.001). The USMLE Step 2 CK score could be estimated from the COMLEX-USA Level 2-CE score using the equation: USMLE Step 2 CK = 0.126(COMLEX-USA Level 1 score) + 163.5. In this model, the standard error of the estimate was 9.1, with a model R^2^ of 0.64.

**Figure 1:** Scatterplot of COMLEX-USA Level 2-CE and USMLE Step 2 CK scores for the 340 students in the study. CE: Clinical Evaluation; CK: Clinical Knowledge; COMLEX-USA: Comprehensive Osteopathic Medical Licensing Examination; USMLE: United States Medical Licensing Examination

## Discussion

Here, we present the association between COMLEX-USA Level 2-CE and USMLE Step 2 CK scores among 340 students from a single osteopathic medical school, the largest in the country, who took both examinations from May 2020 to April 2021. There was a relatively positive linear relationship between performance on these exams, with variation in COMLEX-USA scores explaining approximately 64% of the variation in USMLE Step 2 CK performance, and every one-point increase in COMLEX-USA Level 2-CE score corresponding to a 0.13-point increase in USMLE Step 2 CK score. This linear relationship is similar to the relationship between USMLE Step 1 and COMLEX-USA Level 1 scores from students at the same institution, in which a one-point increase in COMLEX-USA Level 1 was associated with a 0.15-point increase in USMLE Step 1 (standard error = 11.5; model R^2^ = 0.56) [13].

These data fill an important knowledge gap. Although numerous studies have explored the relationship between COMLEX-USA Level 1 and USMLE Step 1 scores, few have evaluated the association between scores on Level 2-CE and Step 2 CK, with each having important limitations. In 2010, Chick et al. [7] reported data from 241 osteopathic applicants to 23 internal medicine programs who took the COMLEX-USA Level 2-CE and USMLE Step 2 CK examinations between 2001 and 2006. However, in the years since, both examinations have undergone significant evolution in their content and format as questions stems are now much longer, buzz words have been heavily redacted, and the content scope continues to evolve [22,23]. Additionally, though a linear association was described (R^2^ = 0.62), the authors did not report the slope or intercept of their regression equation, making it difficult for a given student to predict his or her performance. More recently, Kane et al. [8] evaluated Level 2-CE and Step 2 CK performance among 356 applicants to an emergency medicine residency program from 2006 to 2013, and Russman et al. [10] evaluated 72 applicants to an obstetrics and gynecology program from 2010 to 2014. These studies found a reasonable correlation between COMLEX-USA Level 2-CE and USMLE Step 2 CK scores, with R^2^ values of 0.52 and 0.49, respectively. Although these studies included some students who took these licensing examinations within the past decade, both included only applicants to a single residency program, and only Russman et al. reported a full regression equation (USMLE Step 2 CK = 0.16(COMLEX-USA Level 2-CE) + 134.1) [10].

The contemporary data reported here may be helpful to osteopathic medical students and their advisors in considering whether to take the USMLE Step 2 CK examination. While a high Step 2 CK score may enhance a student’s residency application, a low score or an exam failure is unlikely to do so. Before electing to take an expensive examination that is not required for graduation or licensure, applicants and their advisors may wish to consider the likelihood of achieving a beneficial score against the risk of a harmful one.

The findings here may also be useful to residency program directors in evaluating osteopathic applicants. Even after the realization in 2020 of a single accreditation system [24] and the recommendation that COMLEX-USA and USMLE scores be treated equally [25], many residency program directors still do not have the same comfort in interpreting COMLEX-USA scores as they do scores from the USMLE. Although the National Board of Osteopathic Medical Examiners publishes percentiles for COMLEX-USA performance [26], this information only allows programs to evaluate how osteopathic applicants compare to each other, while USMLE scores can be used as a common measuring stick to directly compare MD and DO applicants. The simple fact is that the majority of allopathic programs are more comfortable evaluating the USMLE and not COMLEX and there is precedent for osteopathic students to take the USMLE and not the other way around. Although neither exam is perfect at evaluating resident performance, there is data on both sides that show a positive correlation between success in COMLEX and USMLE and residency performance [27,28]. It is also unclear which examination better predicts residency outcomes as, to our knowledge, no studies exist. It might be that COMLEX-USA is a better predictor than USMLE, but one problem is that, although osteopathic students are eligible to take the USMLE, allopathic students are excluded from taking COMLEX-USA. The regression equation provided here may provide some middle ground: by inputting an applicant’s COMLEX-USA Level 2-CE score, a program director could obtain a point estimate of the applicant’s most likely USMLE Step 2 CK score.

This work has many strengths. It is the most recent study in the last 10 years that has evaluated the association between COMLEX-USA Level 2-CE and USMLE Step 2 CK scores using recent score data and includes a large sample of students from the largest medical school in the country. With USMLE Step 2 CK scores likely to increase in importance after the transition to pass/fail score reporting for USMLE Step 1, this work provides data that will be useful to osteopathic medical students and their faculty advisors, as well as residency program directors.

Nonetheless, there are important limitations to the findings reported here. First, there are important differences in content between the COMLEX-USA Level 2-CE and USMLE Step CK examinations. While the basic concepts, disease pathology, and treatments are standardized and uniform between the two exams based on the Blueprints of each examination [29,30], the largest obvious difference is that COMLEX places a large emphasis on Osteopathic Principles and Practice which is not tested on the USMLE. It must be emphasized that it is impossible to truly “convert” scores from one exam to another. However, our data show that despite these differences, examinee performance on these examinations is highly correlated.

Second, the equation here is derived from students at a single osteopathic medical school. Overall, 62% of LECOM students took both the COMLEX-USA Level 2-CE and the USMLE Step 2 CK exams, but there were significant differences in test performance among students who chose to take the USMLE and those who did not. From our data, it cannot be determined why some students chose to take USMLE Step 2 CK and some did not, but reasons likely relate to the applicants’ perceived competitiveness and the requirements of the programs to which they intend to apply. Importantly, however, students who chose to take USMLE Step 2 CK had higher performance on COMLEX-USA Level 2-CE than those who took only that test. Based on the data collected, if a larger portion of osteopathic students decided to take the USMLE Step 2 CK, their performance could differ systematically from the performance of the group in whom the regression equation was derived. Common reasons for this are likely explained by the overall competitiveness of the students taking both exams, as well as the specialties chosen by the students taking both exams. The more competitive osteopathic students applying for specialties such as anesthesiology or surgery are more likely to have higher GPAs and COMLEX-USA Level 1 scores than those applying to primary care specialties such as internal medicine and family medicine. Moreover, because these data were obtained in 2020-2021, these students had their medical education disrupted by the novel coronavirus disease 2019 pandemic. Extrapolating these results to populations that systematically differ from the study population may influence the accuracy of the prediction equation. However, in reporting our full linear regression model, we make it possible for other investigators to prospectively validate our findings in other populations.

Third, our analysis was limited only to scores on the USMLE and COMLEX-USA examinations, which were obtained and analyzed in a de-identified format. Other variables that might impact test performance, such as previous standardized tests, dedicated preparation time, or the use of particular test preparation resources, were not considered.

Fourth, the confidence interval for a point estimate derived from our equation is wide: the standard error was 9.1 points. Yet, any prediction of USMLE performance will necessarily be limited by the inherent imprecision of the test itself: the USMLE Step 2 CK examination has a standard error of measurement of approximately six points [31]. In other words, if examinees were tested repeatedly, using different sets of items covering similar content, 95% of their scores would fall within a 24-point range for the examinee’s Step 2 CK score.

## Conclusions

A linear relationship exists between osteopathic medical student performance on the COMLEX-USA Level 2-CE and the USMLE Step 2 CK examinations. Approximately 64% of the variation in USMLE Step 2 CK scores is explained by variation in COMLEX-USA Level 2-CE performance, and every one-point increase in COMLEX-USA Level 2-CE is associated with a 0.13-point increase in USMLE Step 2 CK score. Potential examinees and program directors interested in predicting performance on USMLE Step 2 CK from an individual COMLEX-USA Level 2-CE score can do so using the following equation: USMLE Step 2 CK = 0.13(COMLEX-USA Level 2-CE) + 163.5.
